The article "Development of Advanced Artificial Intelligence and IoT Automation in the Crisis of COVID-19 Detection" was published in 2022. Journal: J Healthc Eng.

# Development of Advanced Artificial Intelligence and IoT Automation in the Crisis of COVID-19 Detection

**DOI:** 10.1155/2022/1987917

**Published:** 2022-03-02

**Authors:** Praveen Kumar Kollu, Kailash Kumar, Pravin R. Kshirsagar, Saiful Islam, Quadri Noorulhasan Naveed, Mohammad Rashid Hussain, Venkatesa Prabhu Sundramurthy

**Affiliations:** ^1^Department of Computer Science and Engineering, Velagapudi Ramakrishna Siddhartha Engineering College, Vijayawada, India; ^2^College of Computing and Informatics, Saudi Electronic University, Riyadh 11673, Saudi Arabia; ^3^Department of Artificial Intelligence, G. H. Raisoni College of Engineering, Nagpur, India; ^4^Department of Civil Engineering, College of Engineering, King Khalid University, Abha 61411, Asir, Saudi Arabia; ^5^College of Computer Science, King Khalid University, Abha 61413, Saudi Arabia; ^6^Center of Excellence for Bioprocess and Biotechnology, Department of Chemical Engineering, College of Biological and Chemical Engineering, Addis Ababa Science and Technology University, Addis Ababa, Ethiopia

## Abstract

Internet of Things (IoT) is a successful area for many industries and academia domains, particularly healthcare is one of the application areas that uses IoT sensors and devices for monitoring. IoT transition replaces contemporary health services with scientific and socioeconomic viewpoints. Since the epidemic began, diverse scientific organizations have been making accelerated efforts to use a wide range of tools to tackle this global challenge and the founders of IoT analytics. Artificial intelligence (AI) plays a key role in measuring, assessing, and diagnosing the risk. It could be used to predict the number of alternate incidents, recovered instances, and casualties, also used for forecasting cases. Within the COVID-19 background, IoT technologies are used to minimize COVID-19 exposure to others by prenatal screening, patient monitoring, and postpatient incident response in specified procedures. In this study, the importance of IoT technology and artificial intelligence in COVID-19 is explored, and the 3 important steps discussed such as the evaluation of networks, implementations, and IoT industries to battle COVID-19, including early detection, quarantine times, and postrecovery activities, are reviewed. In this study, how IoT handles the COVID-19 pandemic at a new level of healthcare is investigated. In this research, the long short-term memory (LSTM) with recurrent neural network (RNN) is used for diagnosis purpose and in particular, its important architecture for the analysis of cough and breathing acoustic characteristics. In comparison with both coughing and respiratory samples, our findings indicate poor accuracy of the voice test.

## 1. Introduction

COVID-19 has been reported as a global epidemic by the World Health Organization (WHO), and it travels out across globe. 8.8 million cases were registered globally on June 30, 2020. With a record of 2.64 million cases and 128 lakhs of accidents, the United States is perhaps the most afflicted country in the region [1–3]. Health practitioners face many challenges such as identify signs, diagnose the condition, and take decisions. To overcome these problems, they use computer programs; they battle to ensure the virus identification, which is successful in this situation. In current trends, AI is a rising innovation; it is close to the intellect of man.

The human brain system illustrates the complex issues, but the lot of concerns increases the cost of solving that issue. AI is capable to concurrently quantify a range of issues and remedies. Many people just assume that AI is just about automation, but it is a computer that imitates human consciousness [4]. IoT connects the people worldwide for transmitting the data to the adjacent devices and systems [5]. The issue is a human who uses some sensors can be tracked regular with automatized devices. Original accusations are written to the framework [6]. IoT device operates with the technology and electronic hardware on the network accessible connected devices for the integrated devices. In recent times, IoT designed a new area of research, specifically in the field of medical services, as a modern subject of study in a broad array of academia and business. IoT development form, i.e., healthcare reform systems combine technical and socioeconomic resources [7]. It progresses from the traditional to much more adapted treatment programs wherein patients could be more easily spotted, managed, and tracked.

IoT is an emerging technology that consists of the set of links provided to interconnects with anything, anywhere, any connection, any device, and any period. IoT technology may affect the whole company range, since every device and entity in the digital Internet network might be identified as having huge benefits. Such benefits often include enhanced connection between services, devices, and systems that go beyond the machine status [8]. IoT delivers suitable solutions to a variety of software and systems. Pollution control, wearables, issues in traffic, defense, intelligent infrastructure, transit, disaster aid, healthcare, and commerce are the examples for IoT. Doctors and community care are one of the most intriguing areas of IoT applications. IoT can generate treatment services such as workout, geriatric therapy, remote monitoring systems, and chronic illness administration.

The emphasis can be made by an IoT framework, integrated with AI. Enhance social protection by using monitoring technologies, image-recognition technology, and the use of AI-enabled software and networks to provide, distribute, trace, and control people's access to the public places [6]. Usually, an IoT health service consists of several server-linked detectors. It provides real-time environmental or user tracking. In an epidemic, AI-assisted detectors can also be used to focus on indicators such as body temperature, respiratory rate, and cough habits of individuals.

A further helpful function might be monitoring people's geolocation. The difference between people could provide helpful info during epidemic of a deadly virus [4]. We will get a fair estimation about how much people share while moving in public spaces using technology like Ethernet.

It is also important to understand the protection and information security extensively during the implementation of certain applications in order to avoid the misuse of confidential data [5]. Authorities may continue to be using these resources and knowledge to continuously observe the actions of individuals after an epidemic. The healthcare sector has long been one of the major areas of application for the IoT. Based on the latest developments in AI and machine learning, eHealth has recently risen to greater heights. The COVID-19 pandemic strategy has provided shudders from several angles across the globe, such as its ability and deliverable, rapid reaction, connected information, and assessment.

The area of eHealth used by IoT and AI to healthcare has mainly become interdisciplinary and offered new horizons to problems during the COVID-19 pandemic [9]. In contrast, technology fields such as IoT and AI have been strongly encouraged to offer rapid and effective medical services, particularly with a view to COVID-19, frequently to automate and facilitate various activities for health professionals.

AI algorithms in particular forecasts play an important role in the study of epidemics. With enormous information on this pandemic, the machine learning methods assist to discover ways to prevent the transmission of the virus from taking prompt action [10]. This search uses the machine learning and deep learning methods to monitor everyday behavior in anticipation of COVID-19' future cross-country accessibility utilizing the official open information source in real-time. These models can predict the near future and help to reduce the harmful consequences of COVID-19. The advent of AI revolutionizes every social and personal sector. AI is designed to behave like a human brain and to mimic its processes of thinking that automate different jobs.

AI is data-driven and makes choices based on the data on which it has been trained. AI is needed to cope with the present epidemic since it has the advantage over the previously mentioned conventional methods. Although AI cannot supplant physicians, it helps them to make diagnostic choices efficient and accurate. Techniques may be used to change the healthcare sector. In pandemic conditions, the healthcare system is overburdened with the enormous number of patient demands, and AI can support them as quickly as practicable with minimal cost for diagnosis and treatment. AI algorithms, such as sensors and cameras, may be readily incorporated into the current infrastructure to automate the contact tracking process. AI helps to do simulations for the prospective medication during the vaccine development process to estimate its efficacy.

The WHO has reported the pivotal symptoms of COVID-19, including body pains, increased heart rate, strong coughing, and severe breathing difficulties [11]. Scientists believe that the respiratory system's audio noises may be identified and examined for the disease's existence. The absurd and stepped-up proliferation of the COVID-19 virus has led to enormous cooperation across many sectors to regulate and prevent the propagation of the virus on a daily basis. In addition, the solution will participate in the fight against COVID-19 in an innovative and the current manner by integrating AI and deep learning algorithms in the digital health district. There have been enormous executions of AI along with the techniques of deep learning (DL), which can be rational during the initial detection and monitoring processes of COVID-19 through the analysis of extracted features of coughing, breathing, and speech using the recurrent neural network (RNN) for coughing, breathing, and speech.

## 2. Review of Literature

Brem et al. [12] infection predictor to reduce the threat of predictive modeling with regard to sustainability variables has been introduced. They also developed to predict the hazards to the effects of chronic and to identify complications by using SVM classifications to identify the health conditions. Wu et al. [13] introduced a methodology for heart disease diagnosis to solve the medical challenges such as irregular heartbeat. To do this, they use the naive Bayesian method. This intelligent device evaluates and classifies data gathering. Rahman et al. [14] computerized improved teaching approach implemented including IoT computers. They used identities to classify the students' intelligibility and standard. This approach helps the students to evaluate without any public health consequences. Javaid et al. [15] suggested a framework to describe the geographic distribution of COVID-19 disease outbreaks.

Bayindir [16] suggested any IoT application to fight COVID-19. Javaid et al. [15] discussed how various 4.0 industries (e.g., IoT and artificial intelligence) might contribute to decrease the disease spread. Mokbel et al. believed that interaction tracking should be the duty of the utilities and offer a largely automated contact tracking design that is not dependent on user participation. Nasajpour et al. [17] discussed various IoT devices in three major phases: diagnosis, isolation, and healing. The application of ML, AI, and other intelligent methods for COVID-19 prognostics is discussed recently.

Dong and Yao [18] discussed about the promising IoT-based approaches to fight COVID-19 that have been developed. They provide a thorough investigation of current IoT systems at various levels, such as perception layers, network layers, and fog and cloud layers. They also explore uses of IoT in the diagnosis of COVID-19 signs. A four-layered architecture is built on the technology by IoT and blockchain to assist combat COVID-19. The chain-based approach for ensuring the confidentiality and security of physiological information exchanged between IoT nodes is suggested. It also includes the several apps designed to identify and trace the proposed approach with COVID-19. IoT's involvement is in the current digital healthcare system. It also discusses the consequences of IoT-generated data that permitted the healthcare system for policy-makers' choices. Additionally, current facilitators and obstacles to IoT-based healthcare are also included.

They identified the capability of the wireless connection and evaluated the network transfer to diagnose the area at greater hazard. They will also obtain greater attempts to monitor the spreading in some areas. Gupta and Johari [6] planned to identify the resource field utilizing IoT sensors including wireless communication technology 802.11 which was an IoT-based control mechanism. They built a modeling approach for tracking the small spaces. The sensors in light lamps have been fixed to track scheduling and the unnecessary use.

Siriwardhana et al. [4] addressed the production and implementation of IoT-based technology to combat the COVID-19 epidemic effectively. In particular, many scenarios and problems are raised, including how 5G and IoT may be candidates for creative technologies in diverse fields to tackle the pandemic. A systematic analysis has likewise been proposed to minimize the contribution made by big technological innovations including such 5G, artificial intelligence, UAV, Internet of Things, and blockchain.

Hussain et al. [5] emphasized using AI to tackle the epidemic COVID-19. This research offered an outline of different cognitive technologies for various types of epidemics dependent on clinical experience. The study classifies the current AI strategies in medical studies analyzes into neural systems, classical vector assistance, and pervasive processing. Last, a thorough explanation was given about the benefits of AI in the fight against related viruses.

Wu et al. [13] suggested a combined protection and health surveillance framework for IoT. The purpose was to increase safety in the open air. The framework contains two layers: one for gathering user information and the other for aggregating information gathered and over the Web. Wearable systems have been used to collect the public safety metrics and consumer health signs.

Afshar et al. [19] claimed that many research studies have been carried out in support of automatic diagnosis and screening of COVID-19. In the eHealth sector, AI can be gripped and pushed to help identify COVID-19 early by monitoring these three major sound systems, including cough, breath, and speech. In addition, pulmonary noises may include many indicators of the health status of human beings that can be identified and treated by the use of machine learning techniques. Consequently, doctors and experts have recently considered detecting COVID-19 from lung noises since before the large epidemic of COVID-19.

## 3. Conceptual Framework

### 3.1. Artificial Intelligence for COVID-19 Pandemic

AI has proven to be a scientific development. It is an incredibly powerful method to solve the COVID-19 epidemic if adequately used [5]. The following are the few present and ability for AI to support the officials in fighting successfully the COVID-19 epidemic:

- Monitoring of illness
- Risk forecasting
- Monitoring of surgical examination
- Healing studies
- Study and simulation of the virus
- Site recognition
- False news for breaking
- Implement the steps to shut down

Many of the above methods are discussed in depth in the following.

#### 3.1.1. Monitoring of Illness

On December 31, 2019, a Toronto-based city health firm, Blue Dot, announced an imminent coronavirus outbreak. The Blue Dot AI system includes various machines learning and natural language processing (NLP) instruments to locate signs of infections that are developing. This ability allows Blue Dot to control the SARS-CoV-2 spread and predict that it would evolve long before pathologists. But this would not go so far as to suggest that there was no human experience to do so as well. Although your model of AI might forecast the epidemic, human knowledge of the model performance remained key.  Figure 1 shows the interfacing of AI for COVID-19 pandemic.

#### 3.1.2. Forecasting of the Risk

An important field of study was the use of prediction techniques to support hospital resource planning. The time-series analysis has been one of the most common methods used to generate short-term demand predictions since it offers thorough treatment for seasonality and serial correlations. For example [16], the prediction of short-term utilization of beds for various time-series techniques and historical average models was assessed [17]. Time-series techniques for predicting occupancy in an urgent ward are analyzed and demonstrated that they can offer meaningful data for up to one week. They exposed that the model generates excellent predictions, but in a crisis, it falls. On a separate line of research [20], patient-level data were used in a computationally expensive model to anticipate the demand at various hospital units.

#### 3.1.3. Medical Diagnosis and Screening

Rapid COVID-19 diagnoses can permit authorities to take appropriate action to restrict the greater dissemination of the infection. Although, the scarcity of reagent kits internationally has complicated the success of huge diagnostic imaging by the officials. Most established AI techniques have been recast, whilst others will be developed to reduce this issue.

#### 3.1.4. Healing Studies

As new, the lack of appropriate virus diagnostic and counseling procedures is one of the largest challenges with SARS-CoV-2. However, AI is known to have an achieve design to accelerate the manufacturing process by evaluating the latest COVID-19 instances as well as ongoing studies into viral infections. A variety of organizations and research laboratories have also used AI to classify new COVID-19 therapies. AI not only can speed things up in clinical trials but can also help to diagnose the established medicines.

#### 3.1.5. Study and Simulation of Virus

Knowing the infection is just the secret to establishing the appropriate cure of COVID-19. Pathogens never replicate on their own, so that they can generate versions of their DNA using cell membranes. For this reason, an infection normally destroys the cell wall through a Keychain system by connecting itself with the host receptors. For most antibody substances, the operational function is to avoid this by removing the cell surface receptors. Therefore, researchers can design the consensus that exists in developing the successful inhibitors.

#### 3.1.6. Site Recognition

The SARS-CoV-2 belongs to the beta-CoV tribe of attention and respect. Genotypes of such diseases usually consist of a combination of populations (bats and rodents). To present, an unexplained element is the biological host that made it easier to relay COVID-19 for humans. To correlate the bacterial vector efficiently and for recognition of differences among recognized viruses, machine learning algorithms have been used. The study proposes that the seasonal influenza species uses the decision tree algorithm. The SARS-CoV-2 can also be expanded to incorporate these versions.

#### 3.1.7. False News for Breaking

Currently, it is unpredictable days since the COVID-19 epidemic have produced some theories and explanations of deception. There has been a lot of disinformation on social networking sites. Technology firms including Google, YouTube, and Facebook have used AI strategies to avoid the dissemination of such false information as well as provide checked facts. Both the networks have sought to filter the material with even the smallest disinformation. In fact, YouTube has put in place tough steps to gather some false video news.

#### 3.1.8. Implement the Steps to Shut Down

A great several nations around the globe are using AI to encourage social dissociations and lock-up initiatives, including China, India, the United States, and the United Kingdom. In China, Baidu has established machine view (CV) operated infra-road monitors to search public areas, making it one of the biggest AI and network companies in the world. These devices not only recognize individuals with elevated physical heat but also distinguish residents who are not adopting the lockdown steps using their built-in face recognition system. A similar CV surveillance system was used to track the public dissociating steps taken by masses in Oxford, England.

### 3.2. Internet of Things Presence in Procedures for COVID-19

IoT offers strategically advanced forum for tackling the COVID-19 epidemic which overcomes the big lock-up difficulties [9]. This system aims to collect up-to-date information and displays the important functions that IoT is used during COVID-19 in the injured individual. IoT is being used to collect the healthcare information from different infectious patients' positions and to handle all the information through virtual management platforms in the first stage. This system enhances information management and coordination of the study. Figures 2 and 3 show interfacing of IoT to tackle the epidemic of COVID-19.

### 3.3. Impact of the COVID-19 Pandemic on the Global Economy

Due to the absence of every clear care plan, the greatest available method of protection against epidemic of COVID-19 was established at the time [5]. Nevertheless, the imperative of social distance forced policy-makers worldwide to implement the lockdowns that have signaled a significant split in the world economy. Both facilities that are nonessential were obliged to close down. It led the supply chain to destroy almost all businesses and thus to hazard losing their homes for people around the world.

#### 3.3.1. Automotive Industry

Due to tight locking policies in many countries of the world, the car sector has undergone huge infrastructure delays to combat the epidemic. With social isolation imposed and people needed to stay at home, the use of vehicles, both commercial and personal, has diminished worldwide. The automobiles affiliated with essential services are the only cars still in use.

#### 3.3.2. Aviation Industry

Atmospheric sector has been hit massively by the COVID-19 epidemic. The affected countries including virtually all states were compelled to both globally and domestically to implement a travel restriction. Critical lines of distribution serving cargo and freight planes are the only operational airways.

#### 3.3.3. Tourism Industry

Since the epidemic of COVID-19, the tourist industry was one of the hardest hit sectors. Tourist industry sales make up to 10% of the worldwide GDP.

#### 3.3.4. Construction Industry

Building businesses are expected to face serious disruptions and setbacks attributable to COVID-19 epidemic in existing ventures. As a result of the strict self-quarantine rules, most building companies will have to suspend their nonessential activities before the epidemic comes to an end. This is expected to lead a massive reprogramming of current programs that could lead to serious damages.

#### 3.3.5. Healthcare and Medical Industry

The epidemic COVID-19 has a major impact globally upon these healthcare services, whereas the overeating induced by lockdown acts and travel restrictions has impacted other industries financially, and the safety sector is far from stagnating. Worldwide clinicians are now experiencing the need for COVID-19 patients to be managed by fans, intensive care units (ICUs), and personal protective equipment's (PPE).

### 3.4. Major Advantages of IoT for Pandemic COVID-19

Alsaeedy and Chong [21] All extremely dangerous patients are properly monitored via the Internet of Things. This technology is used to estimate biometric problems, such as hyperglycemia, pulse rate, and heart infections [22]. IoT is a creative and powerful phase in the fight against the COVID-19 epidemic and may make enormous problems during lockdown. This innovation is helpful in strengthening the infected patient's infinite data as well as other important data.  Figure 4 shows the main advantages of IoT in the battle against COVID-19 pandemics.

### 3.5. Role of IoT Technologies and Tools in COVID-19 Pandemic

COVID-19 has a unique effect on society, and the economy of the effect of this epidemic nowadays has increased the use of numerous new technologies in combination with other technologies such as AI, data management, and cloud. IoT is of tremendous help in this disaster IoTs, utilized for epidemic monitoring. Important IoT, AI, and big data innovations that assist with the COVID-19 problem and the several problems stated in that effort include telemedicine's for the prevention and management of disease, the prevention of outbreaks and the minimization or even stoppage of the transmission of the virus, the use of drones to monitor for isolation, and mask use. For COVID-19, primary IoT applications are the online clinics, remote consultations, fast screenings, and the smart monitoring of sick individuals and virus prediction [21], the real-time monitoring, patient monitoring, rapid diagnosis, patient education, testing and tracking, protection, and surveillance. There are additional concerns of confidentiality and protection related to the use of CR. The function of IoMT in monitoring patients from a distant location, the ordering of medical products, and the use of smaller devices to communicate patient data to the authorities concerned [4] focus on the peripheral system and improve quarantined sufferers for different metrics such as respiratory rate, air rate, and lung sound rate, tracking devices to identify infections and monitoring for remote access and diagnosing COVID-19 patients with mild symptoms and tele-health innovations. The function of IoT-based technologies in COVID-19 and the existing IoT solutions for the fight against COVID-19 were examined in three major stages; they separated IoT solutions into primary prevention, confinement period, and recovery. Each step was also shown using IoT-enabled devices including IoT controls, wearable, drones, robots, and smartphone apps.

Suraksha Kawach is an IoT device that is utilized by the Defense Research and Development Organization (DRDO), India, to monitor corona-affected individuals and to monitor them. This gadget may be used in the arm or knee and is a GSM and GPS device for reliable monitoring in real-time basis. The prototype of Suraksha Kawach gadget is shown in Figure 5(a).

In order to minimize healthcare personnel' danger, thermal sensors are used to monitor COVID-19 patients' body temperature.  Figure 5(b) shows the temperature sensor of the sample. We have got wearable gadgets; next, these sensors measure various parameters such as temperature, heart rate, and pulse rate, and the measurement results may be utilized for action as soon as possible. These devices have an important role in containing COVID-19; the intelligent band is one of the wearable devices, as shown in Figure 5(c).

### 3.6. Techniques Used for Coronavirus Sample Collection

To prevent its fast spread, it is necessary to establish valid and realistic medications to treat SARS-CoV-2 disease in people. The nucleic acid test (NAAT) is recommended by the WHO which perhaps the most important model of SARS-CoV-2 detection for the effective SARS disease. These studies include the use of the nasopharyngeal swab procedure in which the cleaning solution is used in a specimen. This contains a combination of mucus and saliva.

In the event of significant breathing problems, the WHO advises that samples be taken from the nose and throat as well. Such specimens are taken to a specialist lab, where the polymerase chain reduction method is used to measure the existence of viral RNA.  Table 1 provides the various techniques for coronavirus sample collection.

### 3.7. Using Artificial Intelligence to Detect, Respond, and Recover from COVID-19

AI systems observed that the epidemic of an unpredictable form of disease in the Chinese government before the world was ever conscious of the danger faced by the coronavirus (COVID-19). With the disease becoming a global epidemic, AI tools and techniques should be used to encourage actions by policy-makers. Furthermore, the health community and the society are essential to plan and control any step of the crisis: identifying, stopping, reacting to, and recovering and growing of COVID-19.  Figure 6 shows the use of AI to detect, respond, and recover from COVID-19.

### 3.8. AI with IoT in Healthcare to Treatment of COVID-19

Since the main report of the 2019 coronavirus infection (COVID-19) in Wuhan, China, more than 200 countries and locations have been affected worldwide. Science and technology take on an important role in this perplexing battle. For example, as China began reacting to infection, it zeroed on brain research by monitoring polluted ancient times moving sick people, robots to convey food and medicines, automatons to clean open spots, and by watching and transmitting sound communication to the public to urge them to stay at home. Man-made knowledge was widely used to identify the new particles in transit to assist COVID-19. A number of experts uses AI to find new medicines and remedies alongside certain software engineering analysts that focus on the identification of compelling patients via the preparation of a clinical image like *X* beams and CT filters [21].

In any case, computer-based intelligence follows the bands to assist group the isolated rule. Advanced mobile telephones and AI-enhanced heated cameras are being used to recognize fever and tinged people [19]. Nations such as Taiwan have combined the public knowledge based on clinical protection with input from the migration and customs data collection, thereby challenging the travel history and side effects of the COVID-19 patients. In all, AI is used to identify, monitor, and hypothesis flares and helps diagnose the illness.

It is used in the treatment of medical claims. Automobiles and robots are used to transport food and medicines, just as they are used to sanitize public areas. AI helps to create the medicines and COVID-19 antibodies using super PCs [17]. This present study focuses on the use of human-made pushes in the fight against the coronavirus epidemic. It provides an extensive review of the innovative drivers utilized to reduce and conceal the significant impact of the upheaval [5]. The motivation of current study is not only to assess the effect of presented methods but also to suggest their use.

## 4. Research Methodology

The program process entails the primary analyses and checks for modern sensors and intelligent systems. Research designs with AI techniques are designed to define a mechanism that underlies the number of environments in order to overcome the difficulty of the problem. The goal of the project is to explore the various sensing devices to gather the multiple information and utilizes the AI systems mostly on data sources. The key objective of the proposed work is to gather information upon this thermal and breathing level of the COVID-19 instances from various devices in real-time. In the data preprocessing, the recorded actual statistics shall be believed to reduce the error and extreme values from the principal component analysis (PCA). The third phase resulted in classifying the COVID-19 instances into three groups such as SIR, disease prone, affected and resuscitated (SIR). Then, in the fourth stage, the deep, simple RNN (recurrent neural network) predicts COVID-19 with past health data.  Figure 7 shows the flow diagram for detection of COVID-19 using IoT and AI. The four steps of the model suggested are as follows:

- Data accession
- Data accusation
- Systemization
- Forecasting

### 4.1. Recurrent Neural Network

The RNN is a class of the ANN that generates a graph structure for spatial and dynamic characteristics analysis. It assists to modeling the sequence information from transmission systems. The prediction findings are identical to the human brains. The processing of knowledge is clear. Assume an easy and simple given set of data feeding just one neuron. The method provides the performance in a typical neural net by increasing the input with the mass and creates strategies. An RNN returns this performance with the bunch of times. We call timestamp of the period, and the output is entered for the next multiplication of matrices. For illustration, the system consisted of one neuron in the image. The system measures the input/weight mathematical operations and applies nonlinearity with the enabling function. The performance at *t*−1 would be the same. This *o*/*p* is the *i*/*p* of the multiplication of the 2nd matrix.  Figure 8 shows the recurrent neural network.

The proposed system consists of 6 neurons. Two important properties of the ANN are as follows.

- Data entered with the first weight set
- Earlier production for a second weight collection

Notice that the quantities of the listed within the first flow forward which are null, and we have no quality present.

### 4.2. SIR Model

This framework is being implemented by Kermack and McKendrick, and it consists of the various classification COVID-19 situations, including such confirmed, contaminated, and rehabilitation instances. The disease deterministic method (Koike and Morimoto, 2018) is being implemented. The proposed method uses the SIR model as follows:

- Suspected (*S*): patients immediately suspected of disease by others
- Infected (*I*): victims infected through whatever requires
- Victims healed by infection, and patients accused of infection from others (*R*)

The design of the outbreak is mathematically written as follows:

(1) $$\begin{array}{c} \frac{\text{d}s}{\text{d}t}=a-\text{d}s-\lambda i+\beta ,\\ \frac{\text{d}i}{\text{d}t}=\lambda i-\left(d+m\right)i-T\left(i\right),\\ \frac{\text{d}r}{\text{d}t}=mi-\left(d+\beta \right)+T\left(i\right), \end{array}$$

where *a* signifies the number of patients being tested; whereas  *i* represent the relative state constant determined by *a*1,  *a*2, the infection rate *b* parameter calculate is the rate of the victims not healed by loss of resistance, *m* is the normal patient's mortality rate, and *T* is a natural cure for the actual individuals diagnosed.

## 5. Result Analysis and Discussion

The table describes that the total population (sample size) of 227 among that population female population of 85 members and male population size of 135 members and other population size of 7 members and 30 members are below 18 years, between 19 and 30 years are 63 members, between 31 and 59 years are 92 members, and above 60 years are 42 members and 33 members having body temperature below 370°C, and 194 members having the temperature (380°C, 390°C, 400°C), and 123 members are infected with COVID-19, and 123 members are in danger zone; they are having different health abnormalities such as breathing problems.

Figure 9 shows COVID-19 effected cases. Figures 10 and 11 show the problematic cases and nonproblematic cases.  Table 2 provides the forecasting of COVID-19 with the selective analytical aspects.  Table 3 provides the COVID-19 effected cases.  Table 4 provides problematic cases.  Table 5 provides nonproblematic cases.

## 6. Conclusion

The threat of the COVID-19 epidemic is still being faced by the universe that attempts complemented by numerous emerging innovations, including such IoT. These are being made by AI to mitigate their impact. Holding that, we have some recent observations of COVID-19 epidemic as the basis for this study. This study is initiated by an exhaustive analysis of COVID-19, wherein we discuss its medical characteristics, dissemination process, and the detection techniques.

For the population analysis, the SIR disease process is employed to identify the events under suspicion; the information is then fed into an LSTM RNN to estimate the COVID-19 instances with past data contained in the secret layer. The two stable problems in electronic enforcement, which requires adjustment, include confidentiality and faith. The migration of data also appears as an additional obstacle to solve interference and complexity by replacing evolutionary methods.

## Figures and Tables

**Figure 1:** AI for COVID-19 pandemic.

**Figure 2:** IoT tackles the epidemic of COVID-19.

**Figure 3:** Increase IoT phase map to tackle the pandemic of COVID-19.

**Figure 4:** Major advantages of IoT for pandemic COVID-19.

**Figure 5:** (a) Suraksha Kawach device 5. (b) Sensor 5. (c) Smart band.

**Figure 6:** Use of AI to detect, respond, and recover from COVID-19.

**Figure 7:** Flow diagram for detection of COVID-19 using IoT and AI.

**Figure 8:** Recurrent neural network.

**Figure 9:** COVID-19 effected cases.

**Figure 10:** Problematic cases.

**Figure 11:** Nonproblematic cases.

**Table 1:** Various techniques for coronavirus sample collection.

Technique	Analysis
NC	A collection of respiratory secretions from the back of the throat can be used for specific bacterial culture
NS	This approach includes having the breathing tube connected to a syringe, as opposed to nasopharyngeal swab procedure, for the processing of specimens from the nasopharynx
ETA	It is a bottom respiratory screening tool by means of a vertical pipe defined as bronchoscope that extracts the specimen from the lungs
BAL	A fiber-optical bronchoscope is transferred through nasal passage into the bronchoalveolary stress that after initiation of a sterile saline solution, a sample was obtained
Blood test	A pulse in the arm takes a blood sample

**Table 2:** Forecasting of COVID-19 with the selective analytical aspects.

S. no.	Population characteristics	Classification	Frequency bands described
1	Gender	Female	Female = 85
		Male	Male = 135
		Others	Others = 7

2	Age	Below 18	Below 18 = 30
		Between 19 and 30	Between 19 and 30 = 63
		Between 31 and 59	Between 31 and 59 = 92
		Above 60	Above 60 = 42

3	Temperature	Below 37	Below 37 = 33
		Above 38, 39, 40	Above 38, 39, 40 = 194

4	Disease find	COVID-19	COVID-19 = 123
		Others	Others = 104

5	Danger zone	Breathing problem/no breathing problem	Breathing problem = 18 No breathing problem = 105

**Table 3:** COVID-19 effected cases.

COVID-19 effected cases = 123	
Problematic	18
Nonproblematic	105

**Table 4:** Problematic cases.

Problematic cases = 18	
Age	Cases
Above 60	10
30–59	6
18–29	2

**Table 5:** Nonproblematic cases.

Nonproblematic cases = 105	
Age	Cases
Above 60	8
30–59	38
18–29	47
Below 18	12

## Data Availability

The datasets used and/or analyzed during the current study are available from the corresponding author upon request.
